# Study on the Therapeutic Effect of Azithromycin Combined with Glucocorticoid on Pulmonary Function and Inflammatory Response in Children with Pneumonia

**DOI:** 10.1155/2022/5288148

**Published:** 2022-03-27

**Authors:** Qingchun Zhao, Junbo Yang, Yongmei Sheng, Min Zhuang, Min Qi

**Affiliations:** ^1^Department of Pediatrics, Yantaishan Hospital, Yantai 264000, China; ^2^Department of Pediatrics, Jiyang People's Hospital, Jinan 251400, China; ^3^Department of Emergency Medicine, Hiser Medical Group of Qingdao, Qingdao 266033, China; ^4^Department of Endocrinology, Zhangqiu District People's Hospital, Jinan 250200, China; ^5^Department of Clinical Laboratory, The Second Affiliated Hospital of Shandong University of Traditional Chinese Medicine, Jinan 250001, China

## Abstract

**Objective:**

The objective is to explore the efficacy of azithromycin combined with glucocorticoids in the treatment of children with pneumonia and its effect on the inflammatory response.

**Methods:**

A total of 86 children with pneumonia were divided into the experimental group (EG) and the control group (CG). Both groups received conventional treatment, the CG was treated with azithromycin and the EG was additionally treated with glucocorticoid methylprednisolone. The therapeutic effect, disappearance time of clinical symptoms, pulmonary function, inflammatory factors, immune function, quality of life, and adverse reactions were measured in the two groups.

**Results:**

After treatment, compared with CG, the total effective rate was significantly elevated, the disappearance time of various clinical symptoms was earlier, and various pulmonary function indexes were increased in the EG. The interleukin-6 (IL-6), tumor necrosis factor-*α* (TNF-*α*), C reactive protein (CRP), and CD8+ levels were reduced, and CD3+ and CD4+ levels were increased in the EG. The quality-of-life scores were upregulated in the EG. Moreover, there was no significant difference in the incidence of adverse reactions between the two groups.

**Conclusion:**

The combined use of azithromycin and glucocorticoids in the treatment of children with *Mycoplasma pneumoniae* infection has a good curative effect, can significantly improve lung function, restore pulmonary inflammatory indexes to normal, and enhance patients' immune function and improve their quality of life, with fewer adverse reactions and safety.

## 1. Introduction

*Mycoplasma pneumoniae* pneumonia (MPP) is one of the most common respiratory diseases in children, and its prevalence is increasing year by year in recent years, accounting for more than 10% to 30% of the total incidence of childhood pneumonia [1]. Pneumonia is the leading cause of death in children. Studies have shown that there are approximately 120 million cases of pneumonia in children under 5 years of age worldwide, of which 1.3 million are deaths, and most deaths occur in younger age groups [2]. Pneumonia occurs when the normal defense mechanisms of the lower respiratory tract are disrupted and invaded by pathogens. As the ability of the lower respiratory tract to clear pathogens is diminished, the proliferation of pathogens triggers immune and inflammatory processes that eventually lead to the accumulation of various cellular debris and fluids in the alveoli, resulting in increased pulmonary resistance, alveolar collapse, and a mismatch between lung ventilation and reperfusion, resulting in pneumonia-related symptoms. Once the disease is infected, the disease will develop rapidly and spread continuously, which can damage the extrapulmonary system and multiple organs. The general signs of pneumonia are fever, shortness of breath, nasal alar expansion, cough, dyspnea, and decreased oxygen saturation [3–5], which not only cause great pain to children but also adversely affect their normal growth and development. Therefore, it is necessary to strengthen the early correct diagnosis and treatment of Mycoplasma pneumoniae infection in children. At present, most scholars believe that the pathogenesis of Mycoplasma pneumoniae is related to the direct invasion injury and autoimmune reaction injury caused by the secretion of related inflammatory factors after being adsorbed on the respiratory epithelial cells.

Children with pneumonia are usually treated with antibiotics, and depending on the severity of the disease, some require hospitalization and supplemental oxygen. Azithromycin is a macrolide antibiotic [6], which inhibits the synthesis of mycoplasma protein and prevents the normal metabolism of mycoplasma, thus effectively treating pneumonia. However, there are also adverse reactions such as gastrointestinal dysfunction and liver function damage [7], and with the widespread use of azithromycin, azithromycin resistance is not uncommon and has progressed to the point of affecting clinical efficacy. Glucocorticoid is a steroid hormone secreted by the adrenal cortex [8], which can regulate protein biology, fats, and related metabolites, thereby exerting anti-inflammatory and antitoxic effects of drugs, and can be used in the clinical treatment of childhood pneumonia. In order to explore the clinical efficacy of methylprednisolone combined with azithromycin in the treatment of children with MPP, a total of 86 children with MPP received in our hospital were treated with methylprednisolone combined with azithromycin, and the inflammatory response was evaluated to provide a certain clinical reference for the treatment of children with pneumonia.

## 2. Materials and Methods

### 2.1. General Information

A total of 86 children with pneumonia at our hospital from January 2019 to January 2021 were divided into the experimental group (EG) and the control group (CG). EG consists of 26 males and 15 females; aged 2–9 years, mean (5.47 ± 2.25) years; weight 11–34 kg, mean (23.39 ± 6.18) kg; disease duration 1–8 days, mean (4.47 ± 2.25) days. CG consists of 24 males and 19 females; aged 2–10 years, mean (6.00 ± 2.53) years; weight 13–35 kg, mean (24.05 ± 5.78) kg; disease duration 1–6 days, mean (3.56 ± 1.75) days. This study was approved by the medical ethics committee (approval no. 20190324068) of the above hospital.

### 2.2. Inclusion Criteria and Exclusion Criteria

1. Inclusion criteria were as follows: ① *Mycoplasma pneumoniae* was diagnosed according to the reference standard [9], and the children were all positive by cold agglutination test; ② the children aged ≥2 years old; ③ the parents of the children had signed the informed consent; ④ they were treated followed the requirements; ⑤ there were complete medical records
2. Exclusion criteria were as follows: ① combined with other infectious diseases; ② severe liver and kidney insufficiency; ③ combined tumor; ④ allergy to the drug in this study; ⑤ recent treatment with antibiotics and glucocorticoids

### 2.3. Treatment Methods

Both groups received general treatment, including cough relief, maintenance of electrolyte balance, antipyretic, antiasthmatic, and oxygen supply.

The CG was injected with 10 mg/(kg·d) azithromycin (National Pharmaceutical Zhunzi H20050098; CSPC Ouyi Pharmaceutical Co., Ltd.), the frequency of injection was 1 time/d, the course of treatment was 5 days, and then, after a 4-day rest, the same treatment was given. The doses were continuously injected for 3 days, and 1 mg/kg of azithromycin (National Pharmaceutical Zhunzi H20050098; CSPC Ouyi Pharmaceutical Co., Ltd.) was administered orally after 4 days. After continuous use for 3 days, the drug was discontinued for 4 days. Based on the treatment of azithromycin in the CG, the EG was given methylprednisolone sodium succinate (National Pharmaceutical Zhunzi H20010098, Sinopharm Rongsheng Pharmaceutical Co., Ltd.) injection treatment, and the first dose was 2 mg/(kg·d), once a day, and after 3–5 days of treatment, the dose was reduced to 1 mg/(kg·d), and the treatment was continued for 3 days. Both groups were treated for a total of 21 days.

### 2.4. Observation Indicators

1. Evaluation of curative effect: the curative effect was evaluated according to the reference standard [10]. The clinical symptoms disappeared, the body temperature was normal, and the chest X-ray was normal, which means recovery; clinical symptoms basically disappeared, body temperature was normal, and the chest X-ray was basically normal, which was markedly effective; clinical symptoms were improved, and the chest X-ray showed that the lesions did not completely disappear, which was effective; clinical symptoms were not improved or even worsened, which was ineffective. Total effective rate = (cured + markedly effective + effective)/total number of cases × 100%.
2. The disappearance time of clinical symptoms (fever, pulmonary rales, tonsil congestion, cough) in the two groups was counted.
3. Pulmonary function: the forced vital capacity (FVC), forced expiratory volume in 1 second (FEV1), and the percentage of both (FEV1/FVC) were measured using a spirometer (Jester, Japan) in the two groups.
4. 4 ml of venous blood was drawn from the two groups of children and then centrifuged at 3000 r/min for 10 min. Then, the serum was collected, and the IL-6, TNF-*α*, and CRP levels were measured by ELISA kits (Thermo Fisher, USA).
5. The adverse reactions and recurrence rates of the two groups were counted. Adverse reactions mainly included liver dysfunction, gastrointestinal reactions, rash, and diarrhea. The incidence of adverse reactions in the two groups was calculated.
6. The level of immune function indicators: 5 mL of fasting venous blood was drawn from the two groups and centrifuged at 3000 r/min for 10 min. Then, the supernatant was collected for testing. Flow cytometry was used to evaluate the proportions of CD3+, CD4+, and CD8+.
7. Quality of life: the quality of life of the children was evaluated using the Leicester cough questionnaire [11] (LCQ). The LCQ score includes 3 dimensions of social, psychological, and physical, with a total of 19 items and a total of 21 points. The higher the score, the better the quality of life of the child. This was completed by parents and children together, and the evaluation was conducted once before and after treatment.

### 2.5. Statistical Methods

SPSS 20.0 statistical software was used for data processing. Measurement data are expressed as (*x* ± *s*), and enumeration data are expressed as (*n* (%)). *t* test and *x*2 test were used to analyze the measurement data and enumeration data, respectively. *P* < 0.05 means that the difference is statistically significant.

## 3. Results

The therapeutic effects were measured in the two groups.

Compared with CG (78.07%), the total effective rate in the EG (95.35%) was significantly elevated (*P* < 0.05), as shown in Table 1.

### 3.1. Measurement of the Disappearance Time of Clinical Symptoms

The time to disappearance of fever, disappearance of pulmonary rales, disappearance of cough, and disappearance of tonsil congestion in the EG was markedly elevated, relative to that in CG (*P* < 0.05), as shown in Table 2.

### 3.2. Measurement of Pulmonary Function

Compared with the CG, the pulmonary function indexes of FVC, FEV1, and FEV1/FVC in the EG after therapy were significantly increased (^*∗*^*P* < 0.05), as shown in Figures 1(a)–1(c).

### 3.3. Measurement of Inflammatory Factor Levels

Compared with before therapy, the inflammatory response indexes of IL-6, TNF-*α*, and CRP after therapy were decreased. Moreover, the above index in the EG was decreased, when compared to CG (^*∗*^*P* < 0.05), as shown in Figures 2(a)–2(c).

### 3.4. Measurement of Immune Function-Related Indicators

After therapy, the CD8+ levels in the EG were down-regulated (^*∗*^*P* < 0.05), while the CD3+ and CD4+ levels were up-regulated, relative to before therapy. Moreover, compared with CG, the CD3+ and CD4+ levels in the EG were significantly elevated (^*∗*^*P* < 0.05), as shown in Figures 3(a)–3(c).

### 3.5. Measurement of Quality of Life

After therapy, the social, psychological, physical, and total scores were all increased, and the EG increased more significantly, relative to that in CG (*P* < 0.05), as shown in Table 3.

### 3.6. Measurement of Adverse Reactions and Recurrence Rates

The incidence of adverse reactions in the EG and the CG has no significant difference (*P* > 0.05). However, the recurrence rate in the EG was significantly decreased, relative to CG (*P* < 0.05), as shown in Table 4.

## 4. Discussion

Pneumonia in children is a common and frequently occurring disease characterized by severe disease and rapid progression. After a child is ill, in a relatively short period of time, the respiratory function and circulatory function of the child will be impaired or even collapsed, which greatly threatens the health of the child and is also one of the important causes of death from pneumonia in children in recent years. Among them, MPP is mainly caused by *Mycoplasma pneumoniae* respiratory tract infection, which is more common in autumn and more common in children. The onset of *Mycoplasma pneumoniae* in children is relatively slow, and the children are accompanied by symptoms such as fever and cough. Some children will have symptoms of sticky sputum and bloody sputum [12], which has a serious impact on the physical and mental health and quality of life of the children.

Azithromycin, a second-generation semisynthetic macrolide antibiotic with phagocytosis of phagocytic bacteria, is the preferred antibiotic for the treatment of MPP. The mechanism of MPP is to cause nonfatal injury or to bind to the target site continuously, significantly prolonging the recovery time of bacterial growth. In addition, the drug can promote the release and development of bactericides, produce the effect of promoting white blood cells, increase the degree of cell damage, and prolong the repair time [13–16]. However, azithromycin still has the disadvantage of a long treatment course, long-term use of azithromycin may cause liver damage, and early withdrawal may cause recurrence, so the effect of single use is not ideal. *Mycoplasma pneumoniae* infection involves cellular immunity and humoral immunity. Glucocorticoids [17, 18] have highly effective anti-inflammatory and immunomodulatory effects, which can control the phagocytosis and release capacity of inflammatory factors in the shortest time and can gradually improve vascular microcirculation, which provides corresponding support for treatment. Methylprednisolone [19–21] is a commonly used glucocorticoid drug, which can block the immune response of the body, improve the immune response of the body, and continue to hinder the inflammatory substances and cytokines, with good therapeutic effect.

In this study, the treatment effect of the EG was better than that of the CG, indicating that the combined use of azithromycin and methylprednisolone can better exert a broad-spectrum pathogenic inhibitory effect, reduce the time of persistent infection of pathogens, and reduce the damage caused by pneumonia to children. Qiu et al. [22] reported that azithromycin combined with methylprednisolone in the treatment of children with pneumonia can shorten the treatment time and exert a better therapeutic effect, which is consistent with the results in this paper. In addition, the clinical symptoms disappeared in a shorter time in the EG, which is consistent with the study of Ye et al. [23], suggesting that combination therapy can quickly exert therapeutic effect, shorten treatment time, and reduce antibiotic dependence. This present study also displayed that there was no statistically significant difference in the incidence of adverse reactions between the two groups, and the adverse reactions were relatively mild, which may be related to factors such as rapid improvement of the disease, reduced treatment time, and reduced antibiotic use. Sun et al. [24] also reported that the incidence of adverse reactions of glucocorticoids in the treatment of children with pneumonia was significantly lower than that of other drugs, and the safety was good. This present study showed that the disappearance time of clinical symptoms in the EG was shorter than that in the CG. The results suggested that methylprednisolone combined with azithromycin has a significant effect on children with MPP, which can not only effectively prevent severe cases such as congestion and pulmonary edema in children but also have a good effect on improving respiratory ventilation and ventilation in children. The pro-inflammatory cytokine TNF-*α* is an important initiator of inflammatory and bactericidal processes, and in bacterial pneumonia, macrophage-derived TNF-*α* is elevated, leading to the recruitment of inflammatory cells to the site of infection [25]. IL-6 is produced by monocytes and macrophages that are activated during bacterial infection and is the major stimulator of most acute-phase protein production [26]. CRP is an acute-phase protein synthesized by the liver and is mainly produced in response to the stimulation of IL-6 [27]. This paper discovered that the CD8+, CD4+, CD3+, IL-6, TNF-*α*, CRP levels, and quality of life in the two groups were improved compared with before therapy, and the improvement degree of the EG was better than that of the CG. These results suggested that methylprednisolone combined with azithromycin in the treatment of children with MPP can effectively improve clinical symptoms such as fever and cough, shorten the disease, and promote the absorption of lung inflammation, thereby reducing the incidence of adverse reactions, enhancing children's immunity, and improving children's quality of life.

## 5. Conclusion

Azithromycin combined with methylprednisolone has a good therapeutic effect in the treatment of children with pneumonia, which is beneficial to control pediatric diseases, quickly relieve clinical symptoms, improve the inflammatory response, and improve pediatric pulmonary function, and has a certain application value.

## Figures and Tables

**Figure 1:** Measurement of lung function. (a) Detection of FVC in the two groups. (b) Detection of FEV1 in the two groups. (c) Detection of FEV1/FVC in the two groups.

**Figure 2:** Inflammatory factors were detected in the two groups. (a) Detection of IL-6, (b) TNF-*α*, and (c) CRP levels in the two groups.

**Figure 3:** Measurement of immune function-related indicators. (a) Detection of CD3+, (b) CD4+, and (c) CD8+ levels in the two groups.

**Table 1:** Measurement of treatment effects in the two groups (*n* (%)).

Group	*n*	Get well	Significantly effective	Effective	Ineffective	Total efficiency (%)
EG	43	22	11	8	2	41 (95.35)
CG	43	13	16	5	9	34 (79.07)
*X* ^2^						8.387
*P*						0.039

**Table 2:** Measurement of the disappearance time of clinical symptoms (*x* ± *s*).

Group	*N*	Fever	Lung rales	Cough	Tonsil congestion
EG	43	1.88 ± 0.49	3.43 ± 1.77	3.12 ± 0.58	4.34 ± 0.94
CG	43	2.26 ± 0.56	4.11 ± 0.83	3.83 ± 0.63	5.13 ± 1.06
*t*		3.380	3.922	5.457	3.652
*P*		<0.05	<0.05	<0.05	<0.05

**Table 3:** Detection of quality of life scores (*x* ± *s*).

Group	*N*	Time	Society	Psychology
EG	43	Before therapy	1.54 ± 0.27	3.77 ± 0.55
		After therapy	2.73 ± 0.42	6.48 ± 0.68
CG	43	Before therapy	1.56 ± 0.32	3.79 ± 0.58
		After therapy	2.04 ± 0.44	5.44 ± 0.67
*t*			7.503	7.070
*P*			<0.05	<0.05

Group	*N*	Time	Physiological	Total score
EG	43	Before therapy	3.91 ± 0.67	9.66 ± 1.12
		After therapy	6.61 ± 0.63	16.21 ± 2.15
CG	43	Before therapy	3.97 ± 0.70	9.53 ± 1.12
		After therapy	5.62 ± 0.68	13.18 ± 1.56
*t*			7.010	7.492
*P*			<0.05	<0.05

**Table 4:** Detection of adverse reactions and recurrence rates (*n*, %).

Group	*n*	Liver dysfunction	Gastrointestinal reactions	Rash	Diarrhea	Recurrence rate
EG	43	1 (2.33)	1 (2.33)	0 (0.00)	1 (2.33)	2 (4.65)
CG	43	2 (4.65)	1 (2.33)	1 (2.33)	0 (0.00)	9 (20.93)
*X* ^2^		0.345	≦0.001	1.012	1.012	5.108
*P*		>0.05	>0.05	>0.05	>0.05	<0.05

## Data Availability

The datasets used and/or analyzed during the present study are available from the corresponding author on reasonable request.
